The article "Long non-coding RNA SLC2A1-AS1 induced by GLI3 promotes aerobic glycolysis and progression in esophageal squamous cell carcinoma by sponging miR-378a-3p to enhance Glut1 expression" was retracted in 2023. Reasons: errors in the images; duplicated images.

# Long non-coding RNA SLC2A1-AS1 induced by GLI3 promotes aerobic glycolysis and progression in esophageal squamous cell carcinoma by sponging miR-378a-3p to enhance Glut1 expression

**DOI:** 10.1186/s13046-021-02081-8

**Published:** 2021-09-13

**Authors:** Hongtao Liu, Qing Zhang, Yinsen Song, Yibin Hao, Yunxia Cui, Xin Zhang, Xueying Zhang, Yue Qin, Guangzhao Zhu, Feng Wang, Jinghan Dang, Shanshan Ma, Yanting Zhang, Wenna Guo, Shenglei Li, Fangxia Guan, Tianli Fan

**Affiliations:** 1 School of Life Sciences, Zhengzhou University, Zhengzhou, 450001 Henan China; 2 Translational Medicine Research Center, Zhengzhou People’s Hospital, Zhengzhou, 450003 Henan China; 3 Institute of Genomic Medicine, College of Pharmacy, Jinan University, Guangzhou, 510632 Guangdong China; 4 International Cooperative Laboratory of Traditional Chinese Medicine Modernization and Innovative Drug Development of Chinese Ministry of Education (MOE), College of pharmacy, Jinan University, Guangzhou, 510632 Guangdong China; 5 Department of Clinical Medicine, Zhengzhou University, Zhengzhou, 450052 Henan China; 6 Department of Pathology, the First Affiliated Hospital of Zhengzhou University, 40 Daxue Road, Zhengzhou, 450052 Henan China; 7 Department of Pharmacology, School of Basic Medicine, Zhengzhou University, 100 Kexue Road, Zhengzhou, 450001 Henan China

**Keywords:** Esophageal squamous cell carcinoma, SLC2A1-AS1, miR-378a-3p, Glucose transporter 1, Glycolysis

## Abstract

**Background:**

Emerging evidence demonstrates that lncRNAs play pivotal roles in tumor energy metabolism; however, the detailed mechanisms of lncRNAs in the regulation of tumor glycolysis remain largely unknown.

**Methods:**

The expression of SLC2A1-AS1 was investigated by TCGA, GEO dataset and qRT-PCR. The binding of GLI3 to SLC2A1-AS1 promoter was detected by Luciferase Reporter Assay System and Ago2-RIP assay. FISH was performed to determine the localization of SLC2A1-AS1 in ESCC cells. Double Luciferase Report assay was used to investigate the interaction of miR-378a-3p with SLC2A1-AS1 and Glut1. Gain-of-function and Loss-of-function assay were performed to dissect the function of SLC2A1-AS1/miR-378a-3p/Glut1 axis in ESCC progression in vitro and in vivo.

**Results:**

We identified a novel lncRNA SLC2A1-AS1 in ESCC. SLC2A1-AS1 was frequently overexpressed in ESCC tissues and cells, and its overexpression was associated with TNM stage, lymph node metastasis and poor prognosis of ESCC patients. Importantly, GLI3 and SLC2A1-AS1 formed a regulatory feedback loop in ESCC cells. SLC2A1-AS1 promoted cell growth in vitro and in vivo, migration and invasion, and suppressed apoptosis, leading to EMT progression and increased glycolysis in ESCC cells. SLC2A1-AS1 functioned as ceRNA for sponging miR-378a-3p, resulting in Glut1 overexpression in ESCC cells. MiR-378a-3p inhibited cell proliferation and invasion as well as induced apoptosis, resulting in reduced glycolysis, which was partly reversed by SLC2A1-AS1 or Glut1 overexpression in ESCC cells.

**Conclusion:**

SLC2A1-AS1 plays important roles in ESCC development and progression by regulating glycolysis, and SLC2A1-AS1/miR-378a-3p/Glut1 regulatory axis may be a novel therapeutic target in terms of metabolic remodeling of ESCC patients.

**Supplementary Information:**

The online version contains supplementary material available at 10.1186/s13046-021-02081-8.

## Background

Esophageal cancer (ESCA) is the seventh leading cause of cancer-related death in the world, which consists of two histological types, esophageal squamous cell carcinoma (ESCC) and esophageal adenocarcinoma (EAC) [1, 2]. In China, ESCC accounts for 90% of all ESCA types, and mainly distributes in Lin County and An Yang area, Henan province [3]. Although tremendous advances in diagnosis and treatment of ESCC patients, the 5-year survival rate for ESCC patients is quite poor [4, 5], which may be mainly due to diagnosis at an advanced stage, high recurrence and metastasis [6, 7]. Therefore, it is extremely urgent for us to seek for novel prognostic markers and therapeutic targets for ESCC patients.

Tumor cells mainly obtain energy via a high rate of glycolysis for tumor survival, and this metabolic feature is now considered as one of tumor hallmarks [8]. Otto Warburg has verified that tumor cells preferentially uptake glucose as main energy source to produce lactate, even in the present of plentiful oxygen, to support the increased metabolic rate [9], which is well known as “Warburg effect” or “aerobic glycolysis” [10]. The metabolic characteristics is implicated in a series of the alteration of metabolic enzymes, such as glucose transporter 1 (Glut1, also named SLC2A1), hexokinase 2 (HK2), pyruvate kinase type M2 (PKM2) and lactate dehydrogenase A (LDHA) [11–16]. Notably, many transcriptional factors including c-myc, hypoxia inducible factor-1α (HIF-1α), nuclear factor kappa-B (NF-κB) promote tumor lactagenesis by regulating the expressions of metabolic enzymes [17–19]. Recent studies have demonstrated that targeting glycolysis-related pathways may be a novel therapeutic target for a variety of tumors [20–22], which will link many metabolic enzymes involved in glycolysis. Despite tremendous advances in tumor glycolysis, its regulatory mechanisms implicated its metabolic enzymes and transcriptional factors remain to be further identified.

Long non-coding RNAs (lncRNAs) as key regulatory elements of cell biological processes are longer than 200 nucleotides, without protein-coding potential, which is transcribed by RNA polymerase II [23]. LncRNAs are considered to be involved in many biological processes, including gene expression regulation, decoy for transcription factors, competing endogenous RNAs (ceRNAs) and scaffolding, etc. [24, 25]. Increasing reports have demonstrated that lncRNAs widely participate in cell growth, survival, differentiation, apoptosis, invasion and metastasis [26–29]. Recently, lncRNAs have been reported to be tightly associated with tumor glycolysis [30–32], and thus targeting these lncRNAs may be novel therapeutic strategies for a variety of tumors. Recently, SLC2A1-AS1 as a novel lncRNA has been verified to promote tumor proliferation by absorbing miR-508-5p in lung adenocarcinoma (LUAD) [33]. Besides, SLC2A1-AS1 triggered the suppression of Glut1 expression, further resulting in the inhibition of glycolysis of hepatocellular carcinoma (HCC) by competitively binding to transketolase and signal transducer and activator of transcription 3 (STAT3) [34]. Our previous report revealed differential expression of lncRNAs in ESCA [35], and SLC2A1-AS1 was given our exclusive attention due to in the same human chromosome 1 with Glut1, suggesting that it may be implicated in the regulation of glycolysis in ESCA. However, its roles and regulatory mechanisms involved in glycolysis remain elusive.

In the present study, we reported a novel lncRNA SLC2A1-AS1 in ESCC. We found that SLC2A1-AS1 was frequently overexpressed in ESCC tissues and cells, which might be due to the high expression of transcription factor GLI3, and its depletion suppressed ESCC cell growth in vitro and in vivo, migration and invasion as well as glycolysis, and induced cell apoptosis in ESCC cells. Mechanistically, SLC2A1-AS1 sponged miR-378a-3p to enhance the Glut1 expression, which further triggered the increased glycolysis in ESCC. Taken altogether, our current data presented herein suggest that SLC2A1-AS1/miR-378a-3p/Glut1 regulatory axis plays an essential role in ESCC development and progression, and thus targeting the signal axis may be a novel therapeutic target for ESCC patients.

## Materials and methods

### Tissue samples

Sixty cases of ESCC samples and paired normal esophageal epithelial tissues were obtained during surgical resection at the First Affiliated Hospital of Zhengzhou University from 2010 to 2016. Tissue samples confirmed using H&E staining by experienced pathologists were immediately frozen in liquid nitrogen after resection, which was further investigated by quantitative real-time PCR (qRT-PCR), Western blot and immunohistochemistry (IHC). Informed consent of all tissue samples was obtained from each patient and the utilization of tissue samples was approved by the Research and Ethics Committee of Zhengzhou University in this study. Meanwhile, the study methodologies completely conformed to the standards set by the Declaration of Helsinki.

### IHC assay

IHC assay was performed according to previous reports [36]. In brief, tissue slides were fixed using formalin, embedded in paraffin and cut continuously for 4-6 μm. After deparaffinization, rehydration and antigen retrieval using microwave heating in citrate buffer (pH 6.0). Primary antibodies against Glut1 (Abcam, Cambridge, MA, USA) were incubated with tissue sections. After rinsing, the corresponding second antibody was added to tissue slides. Staining signals were developed using DAB reagent. The staining results were evaluated by two excellent pathologists.

### Public database assay

Gene expression profiles from ESCA patients were downloaded from The Cancer Genome Atlas (TCGA) dataset using the GDC data portal (https://portal.gdc.cancer.gov/repository), which was analyzed according to our previous publication [35]. GEO DataSet (GSE111011) was applied to examine the SLC2A1-AS1, GLI3 and Glut1 expression in 7 cases of ESCC patients and 7 cases of paired normal samples, and GSE43732 was utilized to detect the miR-378a-3p expression in 119 cases of ESCC tissues and paired normal tissues. TCGA database from StarBase (ENCORI) (The Encyclopedia of RNA Interactomes) was used to investigate the SLC2A1-AS1, GLI3, miR-378a-3p and Glut1 expression in 162 cases of ESCA patients and 11 cases of normal samples. GSE111011 was performed to analyze the expression of glycolysis-related proteins in 7 cases of ESCC tissues and corresponding normal tissues.

### Cell lines, cell culture and transfection

Human ESCC cell lines including EC9706, TE1, Eca109, KYSE70, KYSE30, KYSE180, KYSE450, KYSE510 and KYSE520 as well as normal esophageal epithelial cell Het-1A were obtained from the Chinese Academy of Sciences Cell Bank, which was maintained in RMPI 1640 medium supplemented with 10% Fetal Bovine Serum (Gibco, Invitrogen, USA) in a humidified incubator harboring 5% CO_2_. GLI3 siRNA #1, 2 and 3, control siRNA (con-siRNA), SLC2A1-AS1 siRNA #1 and 2, negative control (NC) (Supplementary Table 1), pcDNA3.1, pcDNA3.1-SLC2A1-AS1, pcDNA3.1-GLI3, pcDNA3.1-Glut1 (Supplementary Table 2), NC-mimic, miR-378a-3p mimic, NC-inhibitor, miR-378a-3p inhibitor (GenePharma Company, Shanghai, China), control siRNA and Glut1 siRNA (Santa Cruz company, USA) were transfected into EC9706, TE1 and KYSE180 cells by Lipofectamine™ 2000 (Invitrogen Life Technologies, Carslbad, CA, USA) according to manufacturer’s instruction.

### Cell counting Kit-8 (CCK-8) assay for cell proliferation

CCK-8 kit was employed to evaluate cell proliferation in ESCC cells. Briefly, various treatment ESCC cells (EC9706, TE1 and KYSE180 cells) at a density of 2 × 10^3^ cells per well were seeded into 96-well plates. At the indicated time points, CCK-8 (Beyotime Biotech, Haimen, China) was added to corresponding wells according to manufacturer’s protocol, and absorbance value at 450 nm was determined in a microplate reader (Thermo Scientific, Waltham, MA).

### Colony formation

Colony formation was performed to access the cell proliferation ability. Briefly, ESCC cells (1 × 10^3^) with different transfection were added to 6-well plate for 72 h. Then, fresh medium was used to replace the old medium to culture ESCC cells for continuous 10 days. Finally, ESCC cells was fixed using 4% of paraformaldehyde for 1 h and stained with 0.1% crystal violet for 30 min.

### EdU staining assay

EdU staining assay was performed according to manufacturer’s protocol. EC9706, TE1 and KYSE180 cells (6 × 10^3^ cells/well) were seeded into 96-well plate, and then were transfected with NC, SLC2A1-AS1 siRNA, pcDNA3.1 and pcDNA3.1-SLC2A1-AS1 according to manufacturer’s protocol. Cells were labeled with EdU reagent in a final concentration of 50 μM for 2 h. Cells were rinsed using PBS buffer for 5 min. Subsequently, cells was fixed in PBS buffer containing 4% polyformaldehyde for 30 min, and glycine (2 mg/ml) in a volume of 50 μl was added to cells for 5 min. Finally, TritonX-100 in a volume of 100 μl was used for decolorization for 10 min. Regarding Apollo staining, a total of 100 μl of 1 × Apollo staining liquid was applied to each well, and incubated for 30 min. PBS buffer containing 0.5% TritonX-100 in a volume of 100 μl was used for decolorization for 10 min. Finally, DNA staining was performed using 1 × Hoechst33342 according to manufacturer’s instruction. The photo was taken using florescent microscope.

### Migration and invasion assay by Transwell chamber

Cell migration and invasion were investigated by Transwell chamber without or with Matrigel (BD Biosciences, San Diego, CA, USA) according to previous report [37]. Briefly, EC9706, TE1 and KYSE180 cells (1 × 10^5^) were placed in the upper layer of chamber, whereas 20% FBS was added to underlayer of chamber. Subsequently, migratory and invasive cells were fixed using methanol, followed by staining with crystal violet 48 h after transfection. Finally, the number of invasive cells was investigated under the field of 200× magnification.

### Glucose uptake and lactate production assays

Glucose and lactate assay kits (Nanjing Jiancheng Bioengineering Institute, Nanjing, China) were used to determine the glucose consumption and lactate production according to manufacturer’s instructions. All data obtained were normalized to protein quantitative values.

### Subcellular fractionation

Cell nucleus and cytoplasm RNA isolation kit (Beibei, Biotech, Co. Ltd., China) was used to extract the nuclear RNA and cytoplasmic RNA, respectively, according to manufacturer’s instruction, and then were investigated using qRT-PCR (Supplementary Table 3).

### Fluorescence in situ hybridization (FISH)

SLC2A1-AS1 probe (5′-AAAAGCAAGGCTTGGCTCACAA-3′) was synthesized and labeled using Cy3 by GenePharma Company, Shanghai, China. For FISH assay, EC9706, TE1 and KYSE180 cells were grown in 24-well plates with glass cover slips for 24 h. After immobilization and permeabilization, EC9706, TE1 and KYSE180 cells were hybridized with 20 μM Cy3-labeled SLC2A1-AS1 probe, and 6-diamidino-2-phenylindole (DAPI) was used to stain cell nuclei of ESCC cells. The images were observed with a florescent microscope.

### qRT-PCR

Total RNA was isolated by Trizol reagent (Invitrogen) according to the manufacturer’s instructions. For mRNA analysis, qRT-PCR was performed using Power SYBR_ green PCR master mix (Applied Biosystems) on an ABI 7500 series PCR machine Applied Biosystems using the specific primers (Supplementary Table 3). For miR-378a-3p expression assay, total RNA was reverse transcribed using the miScript Reverse Transcription Kit (Qiagen, Valencia, CA). qRT-PCR amplification for miR-378a-3p was performed using the miScript PCR Kit (Qiagen) using the specific primers (Supplementary Table 3). Experiments were normalized to U6.

### Western blot

Total proteins were extracted from ESCC cells using RIPA lysis (Solarbio, Beijing, China) and the concentration of the proteins was measured by Bradford method. The proteins were separated by SDS-PAGE, and then transferred to PVDF membranes (Millipore Corporation, Bedford, MA, USA). The primary antibodies against E-cadherin, N-cadherin, Vimentin, Glut1, HK2, PFKM, PKM, LDHA and β-actin (1: 200 dilution, Abcam, Cambridge, MA, USA) were incubated with PVDF membrane (Roche, Switzerland) overnight at room temperature after blocking with skimmed milk. Subsequently, the secondary antibody (ZSGB-BIO, Guangzhou, China) was added to PVDF membrane. Finally, enhanced chemiluminescence (ECL) reagent (Beyotime, Haimen, China) was utilized to develop the protein signal.

### The detection of luciferase activity

The dual luciferase reporter assay system was conducted to determine the direct interaction of SLC2A1-AS1 and miR-378a-3p as well as miR-378a-3p and Glut1. Recombinant vector pmirGLO-SLC2A1-AS1-wild type (WT) and pmirGLO-SLC2A1-AS1-mutation (MUT) as well as pmirGLO-Glut1-WT and pmirGLO-Glut1-MUT (TSINGKE Biological Technology, Beijing, China, the sequences of WT and MUT attached in Supplementary Table 4) along with miR-378a-3p mimic and NC-mimic were transfected into EC9706, TE1 and KYSE180 cells, respectively. For luciferase assay, pGL3-basic with SLC2A1-AS1 promoter MUT and WT sequences (Supplementary Table 5) combined with pcDNA3.1 or pcDNA3.1-GLI3 were transfected into EC9706, TE1 and KYSE180 cells. The Luciferase activity was determined using the Luciferase Reporter Assay System (Promega, USA) 48 h after transfection according to manufacturer’s instruction.

### RNA immunoprecipitation (RIP)

RIP assay was performed in EC9706, TE1 and KYSE180 cells by using RNA-binding protein immunoprecipitation kit (Millipore company, Billerica, MA, USA) as described previously [38, 39]. Briefly, RIP lysates were prepared from EC9706, TE1 and KYSE180 cells transfected with miR-378a-3p mimic or NC-mimic, and then were subjected to immunoprecipitation using 5 μl of either a normal mouse IgG or 5 μl of Anti-Ago2 antibody and the Mana RIP™ RNA-binding Protein Immunoprecipitation Kit. The mRNA levels of SLC2A1-AS1 and miR-378a-3p enriched on beads was determined by qRT-PCR (Supplementary Table 3).

### In vivo nude mouse model

Four- to six-week old female BALB/c nude mice purchased from Beijing Vital River Laboratory Animal Technology Co.,Ltd. were utilized for the animal experiment. The protocols of animal experiments were approved by the Animal Experiment Administration Committee of Zhengzhou University. For tumorigenesis assay, EC9706 cells (1 × 10^6^ cells/each mouse) were subcutaneously injected into the right flank of nude mice at their back, with 5 mice per group. When tumor volume reached around 100mm^3^, NC, SLC2A1-AS1 siRNA, pcDNA3.1 and pcDNA3.1-SLC2A1-AS1 were used to inject intratumorly into the nude mice (NC and SLC2A1-AS1 siRNA modified by methylation and cholesterol, 2 nM for each mouse; pcDNA3.1 and pcDNA3.1-SLC2A1-AS1 for each mouse with 2.5 μg) twice every week for a total of 4 weeks. Tumor volume was measured twice every week, and tumor growth curve was made using the formula “length×width^2^ × 3.14/6”. The mice were euthanized when the experiment was terminated. The tumor tissues were obtained for the isolation of total RNAs and proteins, qRT-PCR was used to investigate the SLC2A1-AS1 and miR-378a-3p expression, and Western blot was performed to determine the expressions of Glut1, HK2, PFKM, PKM and LDHA proteins.

### Statistical analysis

All experimental data from at least three independent repeats were investigated using GraphPad Prism 6.0 software. Data were presented as mean with standard deviation (SD). The IHC results were examined using chi-square, and survival assay were performed using Log-rank test. For the matched samples, the data was analyzed using Wilcoxon signed rank, and for non-matched samples, the data were compared by Mann-Whitney test. The comparison between two groups was determined using a Student’s t-test, and the comparison of > 3groups was determined using one-way ANOVA, and then Bonferroni test was selected for further statistical assay when datasets contain > 3 groups. A *P* value less than 0.05 was regarded to be statistical significance.

## Results

### SLC2A1-AS1 is upregulated in ESCC and correlated with TNM stage, lymph node metastasis and patients’ prognosis

In this study, we investigated SLC2A1-AS1 expression in ESCA tissues by TCGA database and GEO dataset, the data from TCGA database revealed that SLC2A1-AS1 expression in 162 cases of ESCA samples was markedly higher than that in 11 cases of normal samples (Fig. 1A), with no difference between EAC samples and normal samples (*P* > 0.05) (Fig. 1B), but significance difference exhibited in ESCC samples and normal samples (*P* < 0.0001) (Fig. 1C), suggesting SLC2A1-AS1 may be a novel biomarker for discriminating EAC and ESCC histological types. Further GEO dataset assay demonstrated that SLC2A1-AS1 level in 7 cases of ESCC tissues was significantly higher than that in paired normal esophageal tissues (Fig. 1D). To validate these data, we detected SLC2A1-AS1 expression in 60 cases of ESCC tissues and corresponding normal tissues by qRT-PCR using SLC2A1-AS1 specific primers. The results showed that ESCC tissues displayed higher SLC2A1-AS1 expression than normal tissues (Fig. 1E). Afterwards, FISH assay demonstrated that SLC2A1-AS1 expression in ESCC tissues was dramatically higher than that in normal tissues (Fig. 1F). Meanwhile, we also found the high expression of SLC2A1-AS1 in 4 ESCC cell lines, including EC9706, TE1, KYSE180 and KYSE450 (Fig. 1G). These findings suggest that SLC2A1-AS1 may participate in ESCC development.

**Fig. 1:** SLC2A1-AS1 overexpression is correlated with TNM stage, lymph node metastasis and poor prognosis in ESCC patients. A. StarBase online software assay for SLC2A1-AS1 expression level in 162 cases of ESCA tissues and 11 normal samples. B. TCGA database assay for SLC2A1-AS1 expression level in EAC samples and normal samples. C. TCGA database investigation for SLC2A1-AS1 expression level in ESCC samples and normal samples. D. GEO dataset GSE111011 analysis for SLC2A1-AS1 expression level in 7 cases of ESCC tissues and paired normal tissues. E. qRT-PCR assay for SLC2A1-AS1 expression level in 60 cases of ESCC tissues and corresponding normal tissues. F. Representative images of FISH results regarding the high expression of SLC2A1-AS1 in ESCC tissues. G. The expression of SLC2A1-AS1 was detected by qRT-PCR in a panel of ESCC cells. H. The correlations between SLC2A1-AS1 expression level and clinicopathological features, including gender, sex, smoking, drinking, differentiation degree, tumor size, TNM stage and lymph node metastasis. I. Log-rank test determination for the prognostic value of SLC2A1-AS1 in ESCC patients. Compared to normal tissues or Het-1A cell, *P < 0.05, **P < 0.01, ***P < 0.001 and ****P < 0.0001, indicating statistical significance

To further dissect the role of SLC2A1-AS1 in progression and metastasis of ESCC, we investigated the expression of SLC2A1-AS1 in ESCC patients with diverse clinicopathological features. We found that SLC2A1-AS1 expression was not related to the patients’ gender, age, smoking status, drinking, differentiation degree and tumor size (*P* > 0.05), however, its expression was tightly associated with TNM stage and lymph node metastasis (Fig. 1H). Notably, the survival time of ESCC patients with high SLC2A1-AS1 level was extremely lower than that of ESCC patients with low SLC2A1-AS1 level (*P* < 0.05) (Fig. 1I). These data indicate that SLC2A1-AS1 may be a novel predictor for metastasis and prognosis for ESCC patients.

### Transcriptional factor GLI3 binds to SLC2A1-AS1 promoter and induces its expression in ESCC

To explore possible molecular events implicated in SLC2A1-AS1 high expression in ESCC, UCSC Genome Browser (http://genome.ucsc.edu/) was used to obtain the promoter sequence of SLC2A1-AS1, hTFtarget and JASPAR online software was used to predict the binding site of transcription factors, we found that transcriptional factor GLI3 bound to three potential sites in SLC2A1-AS1 promoter region (Fig. 2A). pGL3-basic with SLC2A1-AS1-promoter-WT or –MUT vectors along with pcDNA3.1 or pcDNA3.1-GLI3 were co-transfected into ESCC cells, the results demonstrated that co-transfection of pcDNA3.1-GLI3 and pGL3-SLC2A1-AS1-promoter-WT extremely enhanced the activity of luciferase in EC9706, TE1 and KYSE180 cells, whereas the other groups displayed no difference (Fig. 2B). To verify the precise interaction site of GLI3 in SLC2A1-AS1 promoter region, three mutation vectors harboring different SLC2A1-AS1 promoter mutation region were constructed, these vectors combined with pcDNA3.1 or pcDNA3.1-GLI3 were co-transfected to ESCC cells, we found that the mutation of site 2 significantly reduced the activity of luciferase in EC9706, TE1 and KYSE180 cells (Fig. 2C), suggesting GLI3 mainly binds to the site2 region of SLC2A1-AS1 promoter.

**Fig. 2:** Transcriptional factor GLI3 binds to the promoter region of SLC2A1-AS1 and manipulates its expression in ESCC cells. A. Three predicted GLI3 binding sites on SLC2A1-AS1 promoter by hTFtarget and JASPAR online software. B and C. The luciferase reporter assay of pGL3-basic SLC2A1-AS1 promoter vector with WT or MUT GLI3 binding sites in EC9706, TE1 and KYSE180 cells transfected with pcDNA3.1 or pcDNA3.1-GLI3 vector. D. StarBase online software assay for GLI3 expression in ESCA tissues. E. TCGA assay for GLI3 expression level in ESCC samples and normal samples. F. GEO dataset GSE111011 assay for GLI3 expression in 7 cases of ESCC tissues and paired normal tissues. G. StarBase online software assay for the correlation between GLI3 expression and SLC2A1-AS1 expression in ESCA samples. H. The detection of GLI3 expression after transfection with GLI3 siRNAs in ESCC cells. I. GLI3 expression assay after transfection with pcDNA3.1-GLI3 vector in ESCC cells. J. GLI3 siRNA markedly downregulates the SLC2A1-AS1 expression in ESCC cells. K. GLI3 overexpression significantly upregulates the SLC2A1-AS1 level in ESCC cells. Compared to pcDNA3.1 or con-siRNA group, **P < 0.01, ***P < 0.001 and ****P < 0.0001, indicating statistical significance

To further elucidate the expression of GLI3 in ESCC, the result of TCGA database revealed that there was no difference in GLI3 expression between ESCA samples and normal samples (Fig. 2D), in which there was no difference between EAC samples and normal samples (Supplementary Fig. 1), however, significant difference was found in ESCC samples and normal samples from TCGA database (Fig. 2E),which was further confirmed by GEO dataset in 7 cases of ESCC tissues and paired normal tissues (Fig. 2F). Further investigation showed that GLI3 expression and SLC2A1-AS1 expression exhibited evidently positive correlation (*P* < 0.0001) (Fig. 2G). To further verify whether GLI3 expression affected the SLC2A1-AS1 expression in ESCC cells, three GLI3 siRNAs designed were transfected to ESCC cells, we found GLI3 siRNA#1, 2 and 3 significantly downregulated the GLI3 expression in EC9706, TE1 and KYSE180 cells (Fig. 2H), whereas pcDNA3.1-GLI3 markedly upregulated the GLI3 expression in EC9706, TE1 and KYSE180 cells (Fig. 2I). Stepwise investigation showed that GLI3 downregulation triggered the decrease of SLC2A1-AS1 expression (Fig. 2J), whereas GLI3 upregulation evoked the increase of SLC2A1-AS1 expression in EC9706, TE1 and KYSE180 cells (Fig. 2K). These findings suggest that GLI3 can bind to the promoter region of SLC2A1-AS1 and manipulate its expression in ESCC cells.

Whether SLC2A1-AS1 affected GLI3 expression in ESCC cells, to this end, we firstly analyzed the possible regulatory correlation of SLC2A1-AS1 by LncACTdb2.0 online software, we found that SLC2A1-AS1 might manipulate the GLI3, VEGFA, RUNX1, etc. (Supplementary Fig. 2A and B), further investigation showed that SLC2A1-AS1 was tightly associated with self-sufficiency in growth signals, evading apoptosis, tissue invasion and metastasis as well as reprogramming energy metabolism (Supplementary Fig. 2C). These findings suggest that SLC2A1-AS1 is widely implicated in tumor progression, metastasis and metabolism, therefore, we further detected several key signaling pathways, which was confirmed to be closely involved in tumor development and progression. We found that SLC2A1-AS1 mainly affected Shh and Wnt signaling pathways. SLC2A1-AS1 downregulation suppressed the expressions of GLI1, GLI3, PTCH1, CD44 and Wnt10A (Supplementary Fig. 2D), whereas SLC1A1-AS1 overexpression enhanced GLI1 and GLI3 expressions in EC9706, TE1 and KYSE180 cells (Supplementary Fig. 2E), in which GLI3 displayed the most significant alteration among all genes, suggesting that SLC2A1-AS1 manipulates GLI3 expression in feedback regulatory manner.

### SLC2A1-AS1 depletion suppresses cell proliferation and induces cell apoptosis in ESCC cells

Sustaining proliferation ability and resisting cell death are two representative tumor hallmarks, which have been verified to be involved in tumor development and progression. Hence, we further investigated the roles of the alteration of SLC2A1-AS1 expression in cell proliferation and cell apoptosis in ESCC cells. Two siRNAs against SLC2A1-AS1 or NC was transfected into EC9706, TE1 and KYSE180 cells, qRT-PCR was used to verify the SLC2A1-AS1 expression. We found that two SLC2A1-AS1 siRNAs were both markedly downregulated the SLC2A1-AS1 expression, in which SLC2A1-AS1 siRNA #2 had the better interference effect (Fig. 3A), whereas pcDNA3.1-SLC2A1-AS1 significantly upregulated the SLC2A1-AS1 expression in EC9706, TE1 and KYSE180 cells (Supplementary Fig. 3A). Subsequently, CCK-8, colony formation and EdU staining was used to assess the proliferation ability of ESCC cells, the results demonstrated that SLC2A1-AS1 downregulation significantly suppressed cell proliferation, reduced colony formation and EdU positive staining cell numbers (Fig. 3B-F), whereas the opposite data was presented after SLC2A1-AS1 overexpression (Supplementary Fig. 3B-F). Further Flow cytometry assay revealed that SLC2A1-AS1 depletion contributed to cell apoptosis (Fig. 3G and H). In contrast, SLC2A1-AS1 overexpression suppressed cell apoptosis (Supplementary Fig. 3G and H). Overall, these data imply that SLC2A1-AS1 functions as an oncogenic lncRNA in ESCC cells.

**Fig. 3:** SLC2A1-AS1 depletion contributes to the suppression of cell proliferation and the induction of cell apoptosis in ESCC cells. A. qRT-PCR was used to determine SLC2A1-AS1 expression following transfection with SLC2A1-AS1 siRNA in ESCC cells. B. CCK-8 assay for cell proliferation at 24 h, 48 h, 72 h and 96 h after transfection with SLC2A1-AS1 siRNA in ESCC cells. C. SLC2A1-AS1 downregulation markedly reduced colony formation in ESCC cells. D. Statistical assay for the number of colony formation in ESCC cells treated with NC or SLC2A1-AS1 siRNA. E. EdU staining assay for EdU-positive cell numbers in ESCC cells treated with NC or SLC2A1-AS1 siRNA. F. Quantitative assay of the ratio of EdU-positive cell numbers in ESCC cells treated with NC or SLC2A1-AS1 siRNA. G. Flow cytometry detection for cell apoptosis in different treatment ESCC cells. H. Quantitative analysis for apoptotic cell numbers in a variety of ESCC cells. Compared to NC group, *P < 0.05, **P < 0.01, ***P < 0.001 and ****P < 0.0001, indicating statistical significance

### SLC2A1-AS1 downregulation inhibits cell migration and invasion accompanying reduced glycolysis in ESCC cells

Metabolic reprogramming has been verified to be involved in tumor progression and metastasis through affecting the expressions of glycolysis-related proteins. Here, we found that SLC2A1-AS1 depletion suppressed cell migration and invasion in ESCC cells (Fig. 4A, B and C), coupled with increased E-cadherin protein expression and reduced N-cadherin and Vimentin protein expressions (Fig. 4D and E), whereas SLC2A1-AS1 overexpression promoted cell migration and invasion in ESCC cells (Supplementary Fig. 4 A, B and C), accompanying reduced E-cadherin protein expression and increased N-cadherin and Vimentin protein expressions (Supplementary Fig. 4 D and E). Further investigation revealed that SLC2A1-AS1 depletion markedly downregulated the expression of Glut1 protein, and suppressed glucose consumption and lactate production (Fig. 4F-I), whereas SLC2A1-AS1 overexpression showed opposite effects (Supplementary Fig. 4 F-I). To further elucidate the underlying mechanisms of glucose and lactate alterations mediated by SLC2A1-AS1, GSE111011 was used to investigate the expressions of glycolysis-related proteins in 7 cases of ESCC tissues and paired normal tissues, we found that Glut1, HK2, PFKM, ALDOA, PKM, GPI, LDHA and PGK1 displayed high expression in ESCC tissues, compared to normal tissues (Fig. 4J), which was also confirmed in ESCC samples, EAC samples and normal samples from TCGA database (Supplementary Fig. 5) as well as in 60 cases of ESCC samples and paired normal samples (Supplementary Fig. 6). To further dissect whether SLC2A1-AS1 affected the above altered glycolysis-related proteins, we selected 4 key proteins (HK2, PFKM, PKM and LDHA) as rate-limiting enzymes of glycolysis. We found that SLC2A1-AS1 downregulation dramatically suppressed the expressions of HK2, PFKM, PKM and LDHA proteins in EC9706, TE1 and KYSE180 cells (Fig. 4 K and L), whereas SLC2A1-AS1 overexpression evidently promoted the expressions of HK2, PFKM, PKM and LDHA in EC9706, TE1 and KYSE180 cells (Supplementary Fig. 4 J and K). These findings suggest that SLC2A1-AS1 depletion suppresses cell migration and invasion by inhibiting EMT progression and glycolysis in ESCC cells.

**Fig. 4:** SLC2A1-AS1 depletion suppresses cell migration and invasion as well as glycolysis in ESCC cells. A. SLC2A1-AS1 downregulation suppresses cell migration and invasion in ESCC cells. B and C. Quantification of migrated cell numbers (B) and invasive cell numbers (C) in a variety of ESCC cells. D. SLC2A1-AS1 depletion suppressed EMT progression in ESCC cells. E. Quantification of E-cadherin, N-cadherin and Vimentin protein relative levels following treatment with NC or SLC2A1-AS1 siRNA. F. SLC2A1-AS1 knockdown suppresses Glut1 protein expression in a panel of ESCC cells. G. Quantification of Glut1 protein relative level following treatment with NC or SLC2A1-AS1 siRNA. H and I. SLC2A1-AS1 downregulation suppressed glucose consumption (H) and lactate production (I) in EC9706, TE1 and KYSE180 cells. J. GEO dataset GSE111011 assay for the expressions of glycolysis-related genes in 7 cases of ESCC samples and paired normal samples. K. SLC2A1-AS1 downregulation suppresses the expressions of glycolysis-related proteins, such as HK2, PFKM, PKM and LDHA, in ESCC cells. L. Quantification of relative expressions of HK2, PFKM, PKM and LDHA after transfection with NC or SLC2A1-AS1 siRNA in EC9706, TE1 and KYSE180 cells. Compared with NC group, *P < 0.05, **P < 0.01, ***P < 0.001 and ****P < 0.0001, indicating statistical significance

### SLC2A1-AS1 acts as a ceRNA and competitively absorbs miR-378a-3p in ESCC cells

To investigate how SLC2A1-AS1 exerts its function in ESCC cells, qRT-PCR assay of SLC2A1-AS1 level in the nucleus and cytoplasm demonstrated that SLC2A1-AS1 was mainly localized in the cytoplasm of ESCC cells (Fig. 5A), which was further confirmed by FISH assay (Fig. 5B). Based on the localization of SLC2A1-AS1, we hypothesized that SLC2A1-AS1 functioned as a ceRNA in ESCC cells, and thus DIANA LncBase Predicted v.2 was utilized to predict the possible binding miRNAs of SLC2A1-AS1. We found that SLC2A1-AS1 harbored the binding sites of miR-378a-3p (Fig. 5C). SLC2A1-AS1 expression displayed the negative correlation with miR-378a-3p in ESCA tissues (Fig. 5D). To test the interaction of SLC2A1-AS1 and miR-378a-3p in ESCC cells, Double Luciferase Report experiment was used to verify their interaction. The results demonstrated that the luciferase intensity was significantly reduced by co-transfecting miR-378a-3p mimic and SLC2A1-AS1 WT, but not in the mutant vector without miR-378a-3p binding site in EC9706, TE1 and KYSE180 cells (Fig. 5E). As a core component of the RNA-induced silencing complex (RISC), Ago2 is involved in miRNA-mediating mRNA destabilization or translational repression, therefore, we further performed RIP assay by anti-Ago2 antibody, we found that SLC2A1-AS1 and miR-378a-3p levels precipitated by anti-Ago2 antibody were dramatically increased compared to IgG group (Fig. 5F and G). Besides, Ago2-RIP assay showed that SLC2A1-AS1 enrichment in miR-378a-3p mimic group was markedly higher than that in NC group (Fig. 5H). Subsequently, we found that SLC2A1-AS1 silencing obviously enhanced miR-378a-3p level (Fig. 5I), whereas SLC2A1-AS1 overexpression dramatically reduced miR-378a-3p level in EC9706, TE1 and KYSE180 cells (Fig. 5J). These data suggest that SLC2A1-AS1 directly regulates miR-378a-3p level in ESCC cells.

**Fig. 5:** SLC2A1-AS1 competitively absorbs miR-378a-3p by ceRNA mechanism in ESCC cells. A. qRT-PR assay of subcellular SLC2A1-AS1 level in the nucleus and cytoplasm of EC9706, TE1 and KYSE180 cells, GAPDH and U6 are employed as endogenous controls. B. Subcellular localization of SLC2A1-AS1 in EC9706, TE1 and KYSE180 cells is investigated by FISH experiment, SLC2A1-AS1 is labeled by Cy3 (red) and nuclei are stained with DAPI (blue). C. The miR-378a-3p binding sites in SLC2A1-AS1 transcript are predicted by DIANA LncBase Predicted v.2. D. The correlation of SLC2A1-AS1 with miR-378a-3p is examined in ESCA samples using the bioinformatics tool StarBase E. Double luciferase report experiment is performed to verify the interaction of SLC2A1-AS1 with miR-378a-3p by co-transfecting pmirGLO-SLC2A1-AS1-WT or pmirGLO-SLC2A1-AS1-MUT along with NC-mimic or miR-378a-3p mimic into ESCC cells, compared to NC group, **P < 0.01 and ****P < 0.0001, indicating statistical significance. F. Fold enrichment of SLC2A1-AS1 by Ago2 antibody or IgG in EC9706, TE1 and KYSE180 cells. G. Fold enrichment of miR-378a-3p by Ago2 antibody or IgG in EC9706, TE1 and KYSE180 cells. H. Enrichment of SLC2A1-AS1 in EC9706, TE1 and KYSE180 cells transfected with NC mimic or miR-378a-3p mimic, (F, G and H, compared to IgG group, ****P < 0.0001, indicating statistical significance). I. SLC2A1-AS1 depletion promotes the expression of miR-378a-3p in EC9706, TE1 and KYSE180 cells compared to NC group, ****P < 0.0001, indicating statistical significance. J. SLC2A1-AS1 overexpression suppresses the expression of miR-378a-3p in EC9706, TE1 and KYSE180 cells, compared to pcDNA3.1, ****P < 0.0001, indicating statistical significance

### The associations of miR-378a-3p and Glut1 expressions with clinicopathological features and Glut1 is a target of miR-378a-3p in ESCC cells

To explore the possible roles of miR-378a-3p and Glut1 in ESCC development and progression, we detected their expressions and investigated their correlations with clinicopathological features. TCGA assay revealed that there was no difference in the miR-378a-3p or miR-378a expressions between ESCC and normal samples or EAC and normal samples (Fig. 6A, Supplementary Fig. 7 A and B), but GEO assay exhibited significant difference in miR-378a-3p expression level between ESCC tissues and normal tissues (Fig. 6B), which was further validated by qRT-PCR in 60 cases of ESCC tissues and paired normal tissues (Fig. 6C) as well as ESCC cells and normal esophageal epithelial cell Het-1A (Fig. 6D). Besides, TCGA and GEO assay demonstrated that Glut1 expression in ESCC and EAC tissues was significantly higher than that in normal tissues (Fig. 6E and F, Supplementary Fig. 8 A and B), which was also confirmed in ESCC cells and normal esophageal epithelial cell Het-1A by Western blot (Fig. 6G and H) as well as in 60 cases of ESCC tissues and paired normal tissues by IHC assay (Fig. 6I, Supplementary Table 6). These findings suggest that low miR-378a-3p or high Glut1 expression may participate in ESCC development and progression.

**Fig. 6:** The expressions of miR-378a-3p and Glut1, and Glut1 is a direct target of miR-378a-3p in ESCC cells. A. The expression of miR-378a-3p is detected in 162 cases of ESCA samples and 11 cases of normal samples by StarBase online software. B. The miR-378a-3p level is investigated in 119 cases of ESCC tissues and paired normal tissues by GEO dataset GSE43732. C. The miR-378a-3p level is determined in 60 cases of ESCC tissues and paired normal tissues by qRT-PCR, compared to normal tissues, ****P < 0.0001, indicating statistical significance. D. The expression of miR-378a-3p is examined by qRT-PCR in a panel of ESCC cells, compared to Het-1A cell, **P < 0.01, ***P < 0.001 and ****P < 0.0001, indicating statistical significance. E. The expression of Glut1 is detected in 162 cases of ESCA samples and 11 cases of normal samples by StarBase online software. F. The Glut1 level is investigated in 7 cases of ESCC tissues and paired normal tissues by GEO Dataset GSE111011. G. Western blot assay for Glut1 protein expression in a panel of ESCC cells and normal esophageal epithelial cell Het-1A. H. Quantification of relative levels of Glut1 in a number of ESCC cells and normal esophageal epithelial cell Het-1A, compared to Het-1A cell, *P < 0.05, **P < 0.01 and ****P < 0.0001, indicating statistical significance. I. IHC assay for Glut1 protein expression in 60 cases of ESCC tissues and paired normal tissues. J. The miR-378a-3p binding sites in Glut1 transcript are predicted by miRDB online software. K. Double luciferase report experiment is carried out to confirm the interaction of Glut1 with miR-378a-3p by co-transfecting pmirGLO-Glut1-WT or pmirGLO-Glut1-MUT as well as NC-mimic or miR-378a-3p mimic into ESCC cells. L. miR-378a-3p mimic upregulates the expression of miR-378a-3p, whereas miR-378a-3p inhibitor downregulates the miR-378a-3p level in ESCC cells. M. miR-378a-3p mimic suppresses the expression of Glut1 protein in ESCC cells. N. The analysis of relative level of Glut1 protein after transfection with NC mimic or miR-378a-3p mimic in ESCC cells. O. miR-378a-3p inhibitor enhances the expression of Glut1 protein in ESCC cells. P. The assay of relative level of Glut1 protein after transfection with NC inhibitor or miR-378a-3p inhibitor in ESCC cells. (K, L and N, compared to NC-mimic or NC-inhibitor, **P < 0.01, ***P < 0.001 and ****P < 0.0001, indicating statistical significance)

To further investigate the associations of miR-378a-3p and Glut1 with clinicopathological features of ESCC patients, GraphPad Prism 8.0 software was used to analyze the their correlations. We found that miR-378a-3p level was not related to ESCC patients’ gender, age, smoking, drinking and differentiation degree (*P* > 0.05), but was closely correlated with tumor size, TNM stage and lymph node metastasis (*P* < 0.05) (Supplementary Table 7). Besides, Glut1 expression was not related to ESCC patients’ gender, age, smoking, drinking and tumor size (*P >* 0.05), but was tightly correlated with differentiation degree, TNM stage and lymph node metastasis (*P <* 0.05) (Supplementary Table 8). These findings suggest that miR-378a-3p and Glut1 may be novel predictors for TNM stage and metastasis of ESCC patients.

To further explore the regulatory role of miR-378a-3p on Glut1 in ESCC cells, miRDB online software was used to predict the target genes of miR-378a-3p. We found that Glut1 had the potential binding sites of miR-378a-3p (Fig. 6J). Further Double Luciferase Report assay revealed that the luciferase intensity was significantly reduced by co-transfecting miR-378a-3p mimic and Glut1 WT, but not in the mutant vector without miR-378a-3p binding site in EC9706, TE1 and KYSE180 cells (Fig. 6K). Subsequently, we detected the miR-378a-3p expression in ESCC cells by tranfecting miR-378a-3p mimic or inhibitor, we found that miR-378a-3p mimic significantly upregulated the level of miR-378a-3p, whereas miR-378a-3p inhibitor markedly downregulated the level of miR-378a-3p in EC9706, TE1 and KYSE180 cells (Fig. 6L). Western blot assay showed that miR-378a-3p mimic dramatically downregulated the expression of Glut1 protein (Fig. 6M and N), whereas miR-378a-3p inhibitor extremely upregulated the expression of Glut1 protein in EC9706, TE1 and KYSE180 cells (Fig. 6O and P). These findings suggest that Glut1 is a direct target of miR-378a-3p in ESCC cells.

### The alterations of proliferation, apoptosis and invasion triggered by miR-378a-3p are reversed by SLC2A1-AS1 and Glut1 overexpression in ESCC cells

To verify whether the biological roles of miR-378a-3p exerted in a SLC2A1-AS1- or Glut1-dependent manner, we transfected ESCC cells using NC mimic, miR-378a-3p mimic, miR-378a-3p mimic plus pcDNA3.1-SLC2A1-AS1 and miR-378a-3p mimic plus pcDNA3.1-Glut1 as well as NC inhibitor, miR-378a-3p inhibitor, miR-378a-3p inhibitor plus SLC2A1-AS1 siRNA and miR-378a-3p inhibitor plus Glut1 siRNA. We found miR-378a-3p mimic suppressed cell proliferation and invasion and increased apoptotic cell numbers (Fig. 7A-E), whereas SLC2A1-AS1 and Glut1 overexpressions recovered in part the effects in ESCC cells (Fig. 7A-E). Conversely, miR-378a-3p inhibitor promoted cell proliferation and invasion and decreased apoptotic cell numbers (Supplementary Fig. 9A-E), whereas SLC2A1-AS1 and Glut1 silencing reversed in part the effects in ESCC cells (Supplementary Fig. 9A-E). These findings revealed that miR-378a-3p functions as tumor suppressor in a SLC2A1-AS1- or Glut1-dependent manner.

**Fig. 7:** miR-378a-3p mimic mediated biological effects is dependent on the SLC2A1-AS1 and Glut1 expression in ESCC cells. A. ESCC cell proliferation was assessed by CCK-8 assay in NC mimic group, miR-378a-3p mimic group, miR-378a-3p plus pcDNA3.1-SLC2A1-AS1 group and miR-378a-3p plus pcDNA3.1-Glut1 group. B. Cell apoptosis was determined by Flow cytometry in the same groups appeared in cell proliferation. C. Quantitative assay of apoptotic cell numbers in different treatment ESCC cells. D. Cell invasion ability was detected using Transwell chamber in various ESCC cells with different groups. E. Quantification of invasive cell numbers in diverse ESCC cells with various groups. F and G. The determination of glucose consumption (F) and lactate production (G) in different groups. H. Western blot assay for HK2, PFKM, PKM and LDHA protein expressions in diverse groups. I. Quantification of the relative levels of HK2, PFKM, PKM and LDHA proteins in different treatment groups. *P < 0.05, **P < 0.01, ***P < 0.001 and ****P < 0.0001 were regarded as statistical significance. J. A proposed scheme of the roles and molecular mechanisms of SLC2A1-AS1 in ESCC progression and glycolysis is presented. Note: 1: NC mimic; 2: miR-378a-3p mimic; 3: miR-378a-3p plus SLC2A1-AS1; 4: miR-378a-3p plus Glut1

Given the links of SLC2A1-AS1 with miR-378a-3p, we put forward to whether miR-378a-3p triggered the alterations of glycolysis in ESCC and whether these changes were also reversed by SLC2A1-AS1 or Glut1. Thus, we investigated the changes of glucose consumption and lactate production as well as glycolysis-related gene expressions. We found that miR-378a-3p mimic reduced glucose consumption, lactate production and the expressions of HK2, PFKM, PKM and LDHA proteins (Fig. 7F-I), whereas SLC2A1-AS1 and Glut1 overexpressions recovered in part the effects (Fig. 7F-I). Conversely, miR-378a-3p inhibitor promoted glucose consumption, lactate production and the expressions of HK2, PFKM, PKM and LDHA proteins (Supplementary Fig. 9F-I), whereas SLC2A1-AS1 and Glut1 silencing exhibited the opposite effects (Supplementary Fig. 9F-I). These findings suggest that SLC2A1-AS1 functions as an oncogenic lncRNA that promoted cell proliferation, migration and invasion as well as glycolysis via SLC2A1-AS1/miR-378a-3p/Glut1 signal axis in ESCC cells (Fig. 7J).

### SLC2A1-AS1 promotes tumorigenesis and glycolysis in vivo in ESCC xenografted nude mice

To verify the roles of SLC2A1-AS1 in ESCC cells xenografted nude mice, chemically modified siRNA and overexpression vector of SLC2A1-AS1 were used to treat the tumor. The tumor growth curve demonstrated that SLC2A1-AS1 knockdown dramatically suppressed tumor growth (Fig. 8A and B), but not affected the body weight of nude mice (Fig. 8C), coupled with SLC2A1-AS1 downregulation and miR-378a-3p upregulation in EC9706 cells xenografted tumor tissues (Fig. 8D and E). Further Western blot assay showed that SLC2A1-AS1 depletion markedly reduced the expressions of Glut1, HK2, PFKM, PKM and LDHA in EC9706 cells xenografted tumor tissues (Fig. 8F and G); whereas SLC2A1-AS1 overexpression displayed the opposite effects on tumor growth (Fig. 8H and I), mice weight (Fig. 8J), the expressions of SLC2A1-AS1 and miR-378a-3p (Fig. 8K and L) as well as the expressions of glycolysis-related proteins (Glut1, HK2, PFKM, PKM and LDHA) (Fig. 8M and N) in EC9706 cells xenografted tumor tissues. These data indicate that SLC2A1-AS1 contributes to ESCC tumorigenesis and glycolysis in vivo.

**Fig. 8:** The downregulation of SLC2A1-AS1 suppresses tumor growth and glycolysis in vivo in EC9706 cells xenografted nude mice. A. Representative image of mice from each group after treatment with chemically modified NC or SLC2A1-AS1 siRNA. B. Tumor volumes are measured twice a week for assessment of therapeutic efficacy of SLC2A1-AS1 siRNA in EC9706 cells xenografted nude mice. C. The body weight of mice is determined twice a week in EC9706 cells xenografted nude mice. D. The expression of SLC2A1-AS1 is detected after the end of therapy by qRT-PCR in tumor tissues of nude mice. E. The miR-378a-3p level is examined at the end of therapy by qRT-PCR in nude mice tumor tissues. F. Western blot assay for the expressions of Glut1, HK2, PFKM, PKM and LDHA proteins in NC group and SLC2A1-AS1 siRNA group, and β-actin is used as loading control. G. Quantification of the relative levels of Glut1, HK2, PFKM, PKM and LDHA proteins in NC group and SLC2A1-AS1 siRNA group. H. Representative image of mice from each group after treatment with 2.5 μg pcDNA3.1 or pcDNA3.1-SLC2A1-AS1. I. Tumor volumes are measured twice a week for assessment of therapeutic efficacy of pcDNA3.1-SLC2A1-AS1 in EC9706 cells xenografted nude mice. J. The body weight of mice is determined twice a week in EC9706 cells xenografted nude mice. K. The expression of SLC2A1-AS1 is detected after the end of therapy by qRT-PCR in tumor tissues of nude mice. L. The miR-378a-3p level is examined at the end of therapy by qRT-PCR in nude mice tumor tissues. M. Western blot assay for the expressions of Glut1, HK2, PFKM, PKM and LDHA proteins in pcDNA3.1 group and pcDNA3.1-SLC2A1-AS1 group, and β-actin is utilized as loading control. N. Quantification of the relative levels of Glut1, HK2, PFKM, PKM and LDHA proteins in pcDNA3.1 group and pcDNA3.1-SLC2A1-AS1 group. Compared to NC group or pcDNA3.1 group, *P < 0.05, **P < 0.01, ***P < 0.001 and ****P < 0.0001 were regarded as statistical significance. Note: 1: NC; 2: SLC2A1-AS1 siRNA; 3: pcDNA3.1; 4: pcDNA3.1-SLC2A1-AS1

## Discussion

Currently, a great number of lncRNAs implicated in tumor progression and glycolysis are rapidly expanding [30, 40]. In this study, we reported a novel lncRNA SLC2A1-AS1 involved in ESCC glycolysis. SLC2A1-AS1 was frequently overexpressed in ESCC tissues and cells, and its overexpression was tightly correlated with TNM stage, lymph node metastasis and poor prognosis of ESCC patients. GLI3 as a transcriptional factor drove the SLC2A1-AS1 expression in ESCC cells, whereas SLC2A1-AS also manipulated the GLI3 expression, which formed an important regulatory feedback loop in ESCC. SLC2A1-AS1 silencing suppressed cell growth in vitro and in vivo, migration and invasion ability, and induced cell apoptosis, coupled with alterations of EMT-related molecules and glycolysis-related proteins. Importantly, SLC2A1-AS1 sponged miR-378a-3p to increase the Glut1 expression, further promoted the expressions of glycolysis-related proteins, which led to ESCC progression and increased glycolysis, and thus targeting SLC2A1-AS1/miR-378a-3p/Glut1 signal axis may be a novel therapeutic target for ESCC patients.

Genome-wide analysis has identified a large number of differential lncRNAs in a number of tumor types. Our previous report has unveiled many differential lncRNAs in ESCA [35]. Based on this study, we focused on SLC2A1-AS1 as a novel lncRNA molecule in ESCA. We found SLC2A1-AS1 was highly expressed in ESCC tissues and cells, and its overexpression was tightly correlated with TNM stage, lymph node metastasis and poor prognosis of ESCC patients, which was similar to the study reported in LUAD [33], but was inconsistent with the data previously reported in HCC [34]. These different expression of SLC2A1-AS1 in different tumor types suggest that SLC2A1-AS1 expression may be tumor dependent. Many studies have revealed that transcriptional factors play important regulatory roles in the expressions of many genes. Wang C, et al. found that c-myc bound to the promoter region of PVT1 to enhance the expression of PVT1 in cervical cancer [41]. HIF-1 was identified to directly bind to the promoter region of PDIA3P1, further resulting in its transcription activation in glioma [42]. Notably, the transcription factor activating enhancer binding protein 2 α (TFAP2A) regulated the transcription of SLC2A1-AS1 by directly binding to its promoter region in LUAD cells [33]. To explore the possible regulatory factors of SLC2A1-AS1 in ESCC cells, hTFtarget and JASPAR online software were used to predict the binding sites of transcription factors in the promoter region of SLC2A1-AS1, we found that GLI3 potentially bound to three sites of SLC2A1-AS1 promoter region. At present, GLI3 has been reported to be tightly associated with tumor development and progression [43, 44]. Further investigation revealed that GLI3 bound to the region of SLC2A1-AS1 promoter and promoted its expression in ESCC cells, whereas SLC2A1-AS1 also affected the expression of GLI3, which formed an important regulatory feedback loop in ESCC cells, however, how SLC2A1-AS1 recruited other transcription factors affecting GLI3 expression needs to be further explored.

  Increasing evidence has demonstrated that lncRNAs are implicated in the regulation of biological processes, such as cell proliferation, apoptosis, invasion and metastasis in a multiple of tumors [45, 46], and manipulation of its expression may be a novel therapeutic strategy [47]. In this study, we verified that SLC2A1-AS1 downregulation suppressed tumor growth and glycolysis in vitro and in vivo, decreased migration and invasion and enhanced cell apoptosis, coupled with increased E-cadherin expression and reduced expressions of N-cadherin, Vimentin, HK2, PFKM, PKM and LDHA proteins, and converse data were obtained following SLC2A1-AS1 overexpression. The alterations of these fundamental phenotypes evoked by SLC2A1-AS1 suggest that SLC2A1-AS1 may function as oncogene in ESCC and play an essential role in ESCC glycolysis.

In general, nuclear lncRNAs play the important regulatory roles in chromatin structure and gene transcription [48, 49], whereas cytoplasmic lncRNAs function as ceRNA to control gene expression [50], implying that the function of lncRNAs is dependent on its subcellular localization. Given the complexity and diversity of lncRNA functions in tumor cells, we firstly examined subcellular localization of SLC2A1-AS1 in ESCC cells. We found that SLC2A1-AS1 mainly localized in cytoplasm of ESCC cells by qRT-PCR and FISH. We hypothesized that SLC2A1-AS1 exerted its function via ceRNA mechanism. Our data supported the hypothesis that SLC2A1-AS1 sponged miR-378a-3p in ESCC cells by Double Luciferase Report Assay. Stepwise investigation from Ago2-RIP assay demonstrated that Anti-Ago2 antibody markedly enriched the SLC2A1-AS1 and miR-378a-3p in ESCC cells, notably, when miR-378a-3p was overexpressed, the enrichment of SLC2A1-AS1 was dramatically enhanced, suggesting that SLC2A1-AS1 and miR-378a-3p appeared in the same RISC in ESCC cells. Meanwhile, SLC2A1-AS1 depletion significantly upregulated the miR-378a-3p level, whereas SLC2A1-AS1 overexpression extremely downregulated the miR-378a-3p level in ESCC cells. These findings indicate that SLC2A1-AS1 functions as the sponge of miR-378a-3p to regulate miR-378a-3p expression in ESCC cells.

There is growing evidence that miRNAs are widely deregulated in a number of tumors, highlighting its key regulatory role in onset, growth and metastasis of tumors [51]. Emerging data suggest that miRNAs play essential regulatory roles in different physiological and pathological processes by targeting a majority of mRNAs [52]. At present, miR-378a-3p has been reported to be involved in tumor development, progression and drug resistance by manipulating a series of targeted genes. For example, miR-378 functions as an enhancer of cell growth, cell survival and angiogenesis by targeting SuFu and Fus-1 [53]. MiR-378a-3p has been confirmed to sensitize tumor cells to cisplatin in ovarian cancer by targeting MAPK2/GRB2 [54]. To further unveil the functions of miR-378a-3p in ESCC, we firstly examined the expression of miR-378a-3p in ESCC. We found that miR-378a-3p was frequently downregulated in ESCC tissues and cells by TCGA database, GEO dataset and qRT-PCR, and its expression was tightly associated with tumor size, TNM stage and lymph node metastasis in ESCC patients, suggesting its implication in ESCC development and progression. To uncover its underlying target genes, miRDB database was used to predict the possible downstream target genes. We found that Glut1 was a potential target of miR-378a-3p. To test the prediction, Double Luciferase Report experiment was used to validate it. We confirmed that miR-378a-3p bound to 3′-UTR region of Glut1 to manipulate its expression in ESCC cells. MiR-378a-3p overexpression markedly suppressed the Glut1 expression, whereas miR-378a-3p inhibitor dramatically promoted the Glut1 expression in a panel of ESCC cells. These findings highlight the link of miR-378a-3p with Glut1 in ESCC cells.

Recent investigation revealed that miR-378a-3p was recognized as the pivotal regulator of energy and glucose homeostasis [55], which will enable us to firmly believe that SLC2A1-AS1/miR-378a-3p axis participates in tumor metabolism. Wang Y, et al. verified that Lnc-p23145 bound to the promoter of miR-378a-3p and suppressed the expression of miR-378a-3p, further released the Glut1 expression in oral squamous cell carcinoma, and thus resulting in the acceleration of tumor glycolysis and tumor progression [56]. MiR-378a-3p evoked the metabolic shift by regulating PGC-1β/ERRγ pathway in breast carcinoma [57]. Here, we found miR-378a-3p mimic suppressed cell proliferation and invasion, promoted cell apoptosis, and triggered the decreases of glucose consumption, lactate production as well as glycolysis-related proteins (HK2, PFKM, PKM and LDHA), which was reversed in part by SLC2A1-AS1 and Glut1 overexpression, whereas miR-378a-3p inhibitor exhibited the opposite effects, which was also recovered partly by SLC2A1-AS1 and Glut1 knockdown. Overall, these findings indicate that SLC2A1-AS1/miR-378a-3p/Glut1 may be a key player in ESCC progression and glycolysis.

## Conclusions

In conclusion, SLC2A1-AS1 functions as oncogene in ESCC, and its expression is tightly associated with TNM stage, lymph node metastasis and poor prognosis. Functional and mechanistic assay suggests that SLC2A1-AS1 silencing suppresses cell growth in vitro and in vivo, migration and invasion, and expressions of glycolysis-related proteins by acting as a ceRNA that sponges miR-378a-3p, which will lead to increased Glut1 expression and enhanced glycolysis-related protein expressions. Our current results indicate that SLC2A1-AS1 may play an essential role in driving tumorigenesis, progression and glycolysis, and SLC2A1-AS1/miR-378a-3p/Glut1 signal axis may be a novel therapeutic target for ESCC patients.

## Supplementary Information

**Additional file 1. Supplementary Figs. 1-9.**

**Additional file 2. Supplementary Tables 1-8.**

## Data Availability

The datasets used and/or analyzed during the current study are available from the corresponding author on reasonable request.

## Abbreviations

LncRNAs: Long non-coding RNAs
ESCC: Esophageal squamous cell carcinoma
ESCA: Esophageal cancer
EAC: Esophageal adenocarcinoma
HIF-1α: Hypoxia inducible factor-1α
NF-κB: Nuclear factor kappa-B
Glut1: Glucose transporter 1
HK2: Hexokinase 2
PKM2: Pyruvate kinase type M2
LDHA: Lactate dehydrogenase A
ceRNAs: Competing endogenous RNAs
qRT-PCR: Quantitative real-time PCR
ENCORI: The Encyclopedia of RNA Interactomes
CCK-8: Cell Counting Kit-8
FISH: Fluorescence in situ hybridization
ECL: Enhanced chemiluminescence
RIP: RNA immunoprecipitation
LUAD: Lung adenocarcinoma
HCC: Hepatocellular carcinoma
STAT3: Signal transducer and activator of transcription 3
TFAP2A: Transcription factor activating enhancer binding protein 2 α
